# Review of Measuring Microenvironmental Changes at the Body–Seat Interface and the Relationship between Object Measurement and Subjective Evaluation

**DOI:** 10.3390/s20236715

**Published:** 2020-11-24

**Authors:** Zhuofu Liu, Vincenzo Cascioli, Peter W. McCarthy

**Affiliations:** 1 The Higher Educational Key Laboratory for Measuring and Control Technology and Instrumentations of Heilongjiang Province, Harbin University of Science and Technology, Harbin 150080, China; 2 Murdoch University Chiropractic Clinic, Murdoch University, Murdoch 6150, Australia; V.Cascioli@murdoch.edu.au; 3 Faculty of Life Science and Education, University of South Wales, Treforest, Pontypridd CF37 1DL, UK; peter.mccarthy@southwales.ac.uk

**Keywords:** temperature, relative humidity, pressure, sedentary behaviour, comfort, discomfort

## Abstract

Being seated has increasingly pervaded both working and leisure lifestyles, with development of more comfortable seating surfaces dependent on feedback from subjective questionnaires and design aesthetics. As a consequence, research has become focused on how to objectively resolve factors that might underpin comfort and discomfort. This review summarizes objective methods of measuring the microenvironmental changes at the body–seat interface and examines the relationship between objective measurement and subjective sensation. From the perspective of physical parameters, pressure detection accounted for nearly two thirds (37/54) of the publications, followed by microclimatic information (temperature and relative humidity: 18/54): it is to be noted that one article included both microclimate and pressure measurements and was placed into both categories. In fact, accumulated temperature and relative humidity at the body–seat interface have similarly negative effects on prolonged sitting to that of unrelieved pressure. Another interesting finding was the correlation between objective measurement and subjective evaluation; however, the validity of this may be called into question because of the differences in experiment design between studies.

## 1. Introduction

Although people have been consistently advised not to sit for long durations without breaks [1,2,3,4,5], prolonged sitting has become an inevitable fact of life for some, with the potential to impact everyone (e.g., long-haul flight travel, car passengers during traffic jams and computer gamers). Furthermore, increasing portability of electronic devices (e.g., smartphones, e-readers, tablet PCs) has made it easy for individuals to prolong their working day or enjoy their leisure time in more sedentary activities. Over 20% of commuters choose to continue working while taking public transport to or from the workplace [2], resulting in an extension of their seated working time by up to one working day (7–8 h) a week. To ensure sales, seat designers need to consider the diverse background of end users and the activities they would be expected to perform while seated. The aim, indeed priority, of seat design is to provide users the experience of feeling fit after sitting for prolonged periods [5,6,7,8,9]. Though anthropometry and activities performed whilst seated are believed to have strong influence on the sitting experience, often it is not possible to create saleable seating with accurate information or to predict usage prior to the design process (e.g., classroom chairs usually have the same dimensions though students may vary greatly in terms of anthropometric characteristics) [2,4,5].

The issue of seat design becomes more critical for those individuals (e.g., wheelchair users) who have to spend most of their daily life being seated not out of choice but borne from necessity. In such cases, seat design needs to compensate for a dearth of normal cues, such as skin temperature, moisture and tissue hypoxia, which would usually subconsciously cause people to fidget or move if they the perceived the problem.

Wheelchair users with neurological damage or dysfunction may neither recognize the subconscious cues related to immobility with prolonged skin compression (such as hypoxia, metabolite accumulation, increased temperature, increased relative humidity, changes in the neural feedback), nor be capable of reacting to these cues (such as people with spinal cord injury). Either the person in the wheelchair, or their caregiver, needs to recognize the necessity to regularly move, to ensure the body weight is dispersed through a different contact area on the seat surface. Apart from releasing accumulated pressure between the body and the contact surface, regular movement also allows ventilation of the compressed region, adjusting the microclimate at the body–seat interface in relation to many factors, not least of which include temperature, oxygenation and relative humidity [10,11,12,13,14]. The restoration of blood flow to the affected region reduces the potential for damage to the integrity of the skin and underlying tissues and lowers the risk of pressure ulcer formation [15,16,17].

Increased sedentary behaviour and reduced physical activity can result in a range of chronic diseases such as obesity, type 2 diabetes, high blood pressure and musculoskeletal symptoms [18], as well as the less easily recognized psychological disorders such as depression, anxiety and even schizophrenia [19,20]. However, one physical illness directly related to prolonged sitting is that of the pressure ulcer, which results from persistent mechanical loading on subcutaneous tissues trapped between a contact surface (e.g., seat pan, mattress or backrest) and a bony prominence such as the ischial tuberosities (ITs) or sacrum [21,22]. Although potentially avoidable, the annual expenditure on pressure ulcer diagnosis and treatment has become a heavy financial burden on health care systems. Apart from the financial burden, if not treated effectively (which might not even be possible in some cases), the situation will sadly worsen, eventually resulting in death [6]. According to a 2008–2012 retrospective study, pressure ulcer-related mortality is very high with more than 60,000 deaths in the United States every year [7].

As sedentary behaviour has become so ensconced in contemporary modern society, more and more attention has been paid to the study of sitting comfort. The industrial concept of comfort and discomfort in the seat industry appears different to the commonly accepted nontechnical definitions. Comfort refers to relaxation and well-being [2,7,8], which can easily be influenced by the surrounding environment and external stimuli (e.g., visual appeal and haptic impression) [5,6]. Discomfort, however, tends to be related to tiredness, pain, soreness and numbness and can be the result of defects in design [2,4]. In other words, discomfort and comfort appear to be influenced by different variables and are not necessarily strongly interrelated to each other [3]. Therefore, attenuating the perceived discomfort (such as the reduction of pain) does not necessarily elevate the level of perceived comfort (such as the appearance of pleasure). There is a general acceptance, however, that in order to increase the level of comfort, the level of discomfort has to be reduced [4,7,8].

Traditionally, subjective sensations (sitting comfort and discomfort) are usually evaluated by self-reported questionnaires. However, it is difficult to determine the varying levels of comfort in the same way as it is possible with discomfort [4]. In addition, it appears that large numbers of participants need to be recruited in order to give an unbiased evaluation. Considering the uncertainty of subjective perception, there has been a recent, yet growing, tendency to attempt to develop objective measurement methods to evaluate the sitting comfort or discomfort. Typical objective measures include interface pressure, microclimate changes (temperature and relative humidity), sitting posture assessment, body movement and other vital signs of the body including blood pressure and muscle activity recorded by electromyography (EMG) [4].

Although related topics have been subjected to review, for instance the comfort of passengers using public transport [2] and interface pressure distribution on office chairs [3,4], to the authors’ knowledge, the issue of objectively measuring microenvironmental changes at the body–seat interface and their relationship with subjective evaluations of comfort and discomfort has not yet been addressed in the peer–reviewed literature. Therefore, the aim of this study was to investigate the types of devices used to objectify sitting comfort/discomfort measurement and the physical parameters derived to represent changes at the body–seat contact surface. In addition, some recent “state-of-the-art” techniques (e.g., artificial intelligence and deep learning [9]) have also been included, as it is our opinion that these have potential for future research in this area.

## 2. Materials and Methods

A range of measurement devices and methods have been employed to model the relationship between measurably objective variables and the seated person’s subjective evaluation, in attempts to quantify the extent that the body–seat microenvironment varies while sitting. The search and analysis of the literature reported here were based on objective variables used in such studies (e.g., temperature, relative humidity, movement and pressure) as well as their interaction with any subjective evaluation (e.g., comfort and discomfort). Regarding the subjective elements, several definitions and models of sitting comfort and discomfort have been presented to date [2,3,4,7,8], however, these all tend to use the terms “comfort” and “discomfort”, hence the simple adoption of these two terms in our search protocol was considered adequate to reveal most articles. As shown in Figure 1, the human perceptions of sitting comfort and discomfort appear to be affected by many factors [2,3,4] including seat materials and structures, performed activities (e.g., reading, writing or consulting) and length of time being seated. To reflect objectively the influence of afore-mentioned factors, measurement tools have been employed to monitor microclimate and pressure changes at the body–seat interface.

A systematic search of the literature was conducted consisting of an electronic database search and reference searching. The retrieved sources included medical (PubMed); engineering (IEEE Xplore, EI Village and ACM) and all science (Web of Science and ScienceDirect) electronic databases. Each database was searched in English only, dating from January 2000 to December 2019. The references of all selected articles were also manually reviewed to identify studies that had not been included by the online retrieval search engines. The inclusion and exclusion criteria for the review were developed a priori. To be included in the literature review, the articles needed to:

1. be published in peer-reviewed journals from January 2000 to December 2019;
2. be written in the English language;
3. include objectively measured parameters (using electronic devices) at the body–seat interface;
4. be either cohort studies, cross-sectional studies, case series or case reports; and
5. include human participants (not manikins).

In the literature review, sitting comfort and discomfort are considered to be independent. The following three categorical terminologies were combined by selecting one from each group and searching within titles, key words and abstracts: group I (“chair”, “seat”, “cushion”, “sedentary”, or “sitting”), group II (“comfort” or “discomfort”) and group III (“temperature”, “humidity”, “pressure”, “posture” or “movement”).

All papers found in the literature search were examined (titles, key words and abstracts) to select those considered meeting the inclusion criteria. Articles were excluded if the titles or key words indicated a sole reliance on either environmental impacts (e.g., thermal environment or moisture) or aesthetic perceptions (e.g., comfort or discomfort). If the titles and key words did not provide sufficient information to enable a clear exclusion or inclusion decision, the abstracts would be scrutinized. In addition, papers discussing only the impact of external stimuli (e.g., brightness, vibration, noise and air flow) on sitter’s sensations were also excluded as those influences on sitting were not generated at the sitting interface.

A peer-review process was applied during the full-review stages in which two reviewers participated. An agreement was reached by mutual consent between the reviewers in the few cases of disagreement. Relevant references cited by the selected papers were checked meticulously by screening titles and abstracts (Figure 2). All selected papers were classified into two categories based on the electronic devices used to collect data samples: microclimate (temperature and relative humidity) measurement and pressure measurement (including in-chair movement).

## 3. Results

Studies utilizing pressure measurement accounted for 37/54 of all publications included in this review, while those reporting on the microclimate (temperature or relative humidity) contributed 18/54 (NB one article [15] was reported in both categories).

When studying the publications for each category chronologically, it is interesting to find that most of the research work was published recently. For example, 13 out of 18 papers (72%) based on microclimate measurement were published between 2012 and 2019, demonstrating a slightly greater yet generally similar increment rate to pressure measurement at 24/37 (65%).

### 3.1. Microclimate Measurement

In recent years, due to the increasing recognition of the negative effects of unrelieved heat and moisture on human health, microclimate changes at the user-seat interface have drawn more attention [1,23,24]. As changes in this category were originally considered to be an individual’s physiological sensation (e.g., “I feel hot/wet”), they used to be subjectively evaluated by questionnaires [25]. However, it is difficult to quantify the varying degrees of such perceptions as they are often individual to the subject. The rapid advancement of Micro-Electro-Mechanical System (MEMS) technology and related electronic instruments (e.g., infrared cameras) has made it possible to monitor the microclimatic changes accurately and reliably at the body–seat interface directly (Table 1). Microclimatic changes at the body–seat interface can be described by using two physical parameters: temperature and relative humidity [25]. 

Owing to the size limitation of the early generations of thermal probes, researchers were constrained in relation to how many probes could be used and where to place them without affecting the participants’ comfort directly [36]. As a result, optimal locations were considered to be under ischial tuberosities and thighs [36], based on the assumption that these sites usually accumulated heat and moisture during prolonged sitting. With the rapid improvement of MEMS technology, the chip size and electronic flexibility made it possible to embed an array of sensors inside the cushions [26,27]. As result, a more complete thermal mapping of the contact surface could be constructed by employing imaging algorithms [28]. In order to explore the microclimatic characteristics at the same locations, use of integrated temperature-humidity-sensors has also been reported in several publications [11,31,35,36,37].

Though most of the research work was conducted in simulated conditions (e.g., laboratories or research rooms), some researchers completed the microclimate measurement in real-life situations such as during on-road driving [37]. It is not possible to determine the role that additional lower limb activity, workplace stresses or ventilation may have had impacts on the outcome in such experiments, however, it could be argued that a more realistic appreciation of the seat function may be possible when measurement is made in the workplace.

To choose a cushion suitable for sedentary activities, a variety of materials have been compared including foam, fabric, straps, air cells and gel bubbles. Additionally, Cengiz and colleagues [35,37] examined the performance of different cushion and cover combinations. The conclusion from objective measurement appears consistent to that from subjective evaluation, namely that the more breathable the materials, the greater the perception of comfort the users report [16,38].

### 3.2. Pressure Measurement

Body–seat interface pressure has been widely explored in the study of sitting comfort and discomfort. As a result, a large number of publications have discussed the negative impacts of applying continuously unrelieved pressure on a person’s health (Table 2). As would be expected, the findings are diverse and include: the average pressure [40,41,42], the centre of force [43], the peak pressure [17,42,44] and the pressure distribution at seat pan and back rest [45,46,47]. In addition to simply quoting the pressure, this parameter has also been used to infer in-chair movement or fidgeting [48].

Diversity in the methods of expressing pressure was matched by the variety of choices in measurement point. Specific areas chosen for measurement included: the ischial tuberosity [42,67], bilateral thighs and buttocks [42,72], pressure ratios between different body parts (lumbar/total, lumbar/back, buttock/total, buttock/back) [69] and the backrest contact area [42,44].

Although pressure has been considered an important component in the generation of skin ulcers and there has been a rapid development of material science and computer technology, the number of scientific publications related to sitting related pressure measurement is not great (n = 37). However, this research field is growing rapidly, with publications doubling in the past ten years (between 2010 and 2019: 25/37) in comparison to 2000–2009 (12/37).

Sitting postures show strong associations with interface pressure distribution, which not only affects subjective sensation but also can lead to serious skin integrity problems if not adjusted properly. A number of classification algorithms have been used to distinguish between different sitting postures (Figure 3).

In the process of interface pressure measurement, the most common measurement method uses a commercially available pressure mat constructed in the form of a force sensitive resistor (FSR) matrix, such as that produced by XSensor (XSensor Technology, Alberta, Canada). There are issues with such systems, usually related to calibration and lost data due to regular distortion of the mat which breaks down the FSR matrix. In addition, these mats are subject to a phenomenon referred to as “hammocking”, where the mat does not follow the contours of the seat, instead forming a cover which straddles across small deviations in the seat. Furthermore, specialized hardware platforms are needed as well as software tool kits. Publications were classified in accordance with the number of sensors being used in the pressure measurement (Figure 4). To reduce the complexity and high power consumption of electronic circuits (the inherent property of resistors), Shu et al. [59] proposed a resistance matrix approach (RMA) which identified sensor outputs by solving the resistance matrix equations. Compared with traditional approaches, RMA improved the efficiency and attenuated the complexity by eliminating the redundant components (e.g., external current sources used to prohibit crosstalk noise).

A number of alternative systems have been designed and implemented in the assessment of seating pressure. One such pressure sensitive material is referred to as a “capacitive textile” which is formed of textile-based conductive electrodes placed on both sides of a compressible cushion (e.g., foam) [74]. Foam based spacers can induce hysteresis errors, leading to Meyer et al. [43] employing the Preisach model to improve the measurement accuracy. This method was shown to be capable of resolving and differentiating between different sitting postures.

An electronic textile (eTextile) cushion system was developed by combining a fiber-based yarn and piezoelectric polymer [75,76]. The use of such integrated sensors aims to produce a more comfortable and noninvasive pressure measurement system, being undetectable by the person sitting on it. A problem with this approach is the potential to generate electrical disturbance. Aiming at suppressing the electrical disturbance, a resampling calibration method was proposed by Xu et al. [64] to counter offset, scaling, crosstalk and rotation effects. In addition, the classification accuracy of different sitting postures was improved using a dynamic time-warping algorithm. To enhance the integrity and cover larger areas with a small number of sensors, Ahmad et al. [51] developed a screen-printed piezo-resistive sensor which contains 16 pressure measuring elements. Along with being thin and flexible, the customized sensors exhibited additionally useful electrical characteristics such as high repeatability and reliability (maximum deviation between different sensing elements <8%) [51]. Beyond that, the signal sampling unit was reported to be power efficient and capable of transmitting data to the computer wirelessly. Another merit of this type of piezo-resistive force sensor relates to the relative low expense associated with its manufacture: only half of the cost compared with traditional load cells and force-sensing resistors [40].

## 4. Discussion

This study reviewed and categorized studies that utilized electronic devices to determine measurable parameters at the body–seat interface associated with sitting comfort or discomfort. Publications that did not measure the microenvironmental changes of the contact surface were excluded (e.g., brightness, noise, vibration and air flow as well as aesthetic feelings and anthropometry).

### 4.1. Relationship between Microclimatic Factors, Comfort and Discomfort

Probes [15,29,33], sensors [11,26,28] and infrared thermography [29,30,39] have been employed to investigate microenvironmental changes between the body and the seat surface; however, each has limitations. Some initial research secured the sensor to the skin of the subject, this would create a microenvironment which could prevent the measurement from the microenvironment created between the seat material and skin [35,37]. To avoid the delicate electronic connections of sensors and probes, both are usually embedded in a seat cushion, a procedure which leads to the sensor being subject to measuring limitations caused by insulated properties of the cushion materials [15]. Furthermore, obtrusiveness of probes may directly interfere with the skin blood flow or raise the subjects’ awareness to the presence of the electrodes [28]. An alternative would be to directly image the region, however, to enable cameras to acquire thermal images has required the participants to stand for short periods, which has many effects both on the subject (e.g., physiological redistribution of blood, thus limiting the pooling effect of sitting) and seat surface (potential thermal exchange between the cushion surface and the environment). In more real-life situations, applications of thermal imaging on wheelchair users could result in more problems than benefits, although it could avoid the need for direct contact while measuring.

Although several disparate cushion materials have been compared in terms of rate of temperature increase and cooling speed after prolonged sitting [10,15,29,30,39], it is challenging to give a consistent conclusion on which is the ideal choice for seat products. This indicates that it is critical to take thermal properties of different materials into consideration when manufacturing cushions. Furthermore, thermal outcomes at the contact surface can be influenced by several components including configuration (e.g., foam-fluid hybrid) [31], ventilation (e.g., strap-based) [10] and structure (e.g., honeycomb-structured) [30]. Consequently, it is crucial to study thermal management capacities of different cushions, especially for prolonged sitting usages (e.g., wheelchair cushion).

Before measuring microclimate changes at the body–seat interface, factors that have impact on the outcomes should be considered, such as the surrounding environments (temperature and humidity), on-road traffic and participants’ clothing. As people tend to produce more heat and sweat more easily in hot conditions, studies usually have been conducted in controlled conditions (e.g., air-conditioned laboratories) [35,37]. Furthermore, participants were asked to wear similar or even the same clothing when attending successive trials arranged on different dates.

In addition, experiments [36] have shown that heat begins to accumulate at the body–seat interface as soon as the user sits down. At the first stage (within initial 15 min), temperature increases sharply and then the speed of thermal changes reduces, approaching to and attaining a plateau gradually [36]. Due to this finding [34,36], shorter trial intervals [13,28,29,30,32,34,39] can be applied to evaluate the thermal properties of different cushion materials. By combining some mathematical models and computer algorithms, thermal changes can also be predicted based on the measured information [36]. Several experimental results showed the nonuniform thermal distribution at the body–seat interface [28,34,36], which highlighted the importance of employing more sensors [71,77] while investigating the thermal changes at the contact surface.

Most of the work (14/18) has employed contact sensors to measure microclimate changes at the body–seat interface, with less than a quarter of publications (4/18) [10,29,30,39] using noncontact tools (i.e., infrared cameras) to measure temperature. However, the noncontact measurements required the participants to be transferred from the seat which inevitably led to inaccuracy due to inconsistencies in the emission of heat. Moreover, thermography is not able to continuously monitor the thermal changes at the body–seat interface.

In terms of studying relative humidity characteristics at the contact surface, compared to temperature measurement there has been little. One possible reason behind this phenomenon might be that the risk of increased moisture on skin damage has been neglected [13]. In fact, accumulated moisture deteriorates the epithelial and subcutaneous tissues and eventually leads to tissue necrosis resulting in pressure ulcers [1]. However, the assessment of relative humidity is not free of complications. Unlike temperature changes at the contact surface, an abrupt relative humidity increase can be seen during the initial contact at the seat surface when a person sits down. This was found to be an artefact caused by moisture from a warmer environment interacting with a colder sensor [26]. In other words, there is a transient impulse response induced during the initial process of sitting down. Unlike the temperature showing significant difference among different materials, relative humidity had no consistent performance which indicates one should be cautious when using relative humidity as a physical factor to study at enclosed interfaces, especially where temperature changes are occurring [13,31]. The combination of relative humidity sensor and temperature sensor on the same structure might help to reduce this artifact in the future and make the relative humidity changes more consistent and reliable.

Although only seven out of 18 publications compared the measured data (temperature and relative humidity information) with questionnaire outputs, the consistency indicates that the objective measurement would be a reliable technique to detect microclimatic changes at the body–seat interface.

### 4.2. Relationship between Interface Pressure, Comfort and Discomfort

Pressure mapping has been widely used to objectively assess and monitor pressure changes at the body–seat interface as accumulated forces (focused or asymmetrical tissue loading) negatively impact the subcutaneous tissues and may lead to discomfort and skin diseases (such as pressure ulcer) in the worst conditions.

In terms of pressure measurement, a number of commercially available products exist, such as the Tekscan (Tekscan Co., South Boston, MA, USA) and XSensor (XSENSOR Technology Co., Calgary, Alberta, Canada) system. These pressure mapping systems have large “sensor” arrays [9,45] being based on a matrix of interconnected piezoresistors [52]. Additional conditioning circuits are necessary to coordinate such a large amount of piezoresistive sensors, resulting in issues related to both reliability and stability of the piezoresistive sensors when used in harsh environments [15,55] or repetitively. Indeed, it is our experience that frequent regular recalibration is advisable in order to ensure reliable measurements. As mentioned above, these sensors and their interlinked circuits can be affected by the environment (e.g., temperature) and the parameter they are measuring (pressure). Prolonged exposure to pressures can lead to creep in the output, furthermore, unloading or reduced loading during prolonged pressurization is associated with hysteresis [54,56].

To illustrate the characteristics of interface pressure, directly measured data were represented in various parameters, including the mean backrest pressure [44,78,79,80], the maximal backrest pressure [44], the seat pan contact area [44], the mean seat pan pressure [44], the maximal seat pan pressure [44,46] and maximum and mean buttocks and back support pressure [72]. By converting the measured pressure values into other variables, some researchers investigated the changes at the contact interface using the pressure distribution pattern over time [80], average contact area [67] and ICM [48,73]. Combining with image processing technique, Xu et al. [64] located the boundary of pressure maps and analysed the radius between sensor elements to the pressure centre.

However, most of the pressure measurements were carried out in simulated conditions including laboratories or research rooms, the exceptions being a small number that were conducted in real working conditions [41,49,70,81]. As the performed tasks have an impact on the pressure distribution [82], it appears necessary to measure pressure in real working/living conditions [83,84,85]. Both Bontrup et al. [49] and Zemp et al. [41] studied working sitting behaviours, of call-centre employees and office workers, respectively. These two independent research groups reported that both sitting positions and body movements were associated with the activities being performed. The derived parameters included mean number of movements, mean number of positional changes per working hour, mean time period of stable sitting and percentage of transient periods during the whole working period.

During an on-road driving trial [70], interface pressure exhibited weak correlation with subjective discomfort whereas the traffic situations and environmental changes played more vital roles. The main difference between office work and vehicle driving is the activity: driving a car requires a fixed (asymmetric) body posture with hands on the steering wheel and one foot on the accelerator while working in office allows individuals to adjust the chair, desk, screen and keyboard as well as body posture. This indicates that the preferred sitting position is strongly dependent on the task being undertaken and caution should be taken when interpreting data from different sitting conditions [2,3,4].

Based on experimental data of six short-term (15–20 min) driving sessions, Kyung and Nussbaum [67] showed that the relationship between pressure measurement and sitting comfort/discomfort was associated with exposure time. Although discomfort is attributable to longer sitting durations, Fasulo et al. [50] found there were no obvious changes regarding peak pressure and average pressure values during sedentary activities. In addition, discomfort appears to be regional in so much as different body parts showed different levels of discomfort after prolonged sitting, for example Porter et al. [70] observed an increase in discomfort in the back, buttocks and thighs over time (after a 135-min drive). This suggests that subjective assessments should be considered in more detail than simply using an overall score, as increasing regional assessment might help determine where change needs to be made.

Though the relationship between the contact surface pressure and subjectively perceived comfort/discomfort has been investigated previously [2,4], there is a lack of consistency in terms of those postures considered optimal for sitting comfort. Fasulo et al. [50] pointed out that continuous body movements could release the pressure and increase lower body comfort, while Cascioli et al. [48] found that ICM [73] was a strong indicator of sitting discomfort.

There appears to be many factors that can affect sitting comfort/discomfort, such as seat pitch, legroom space and anthropometry. Passengers prefer to sit next to a vacant seat during the long-haul air travel [83]. Moreover, seats with good views and head or footrests reduce the feeling of discomfort [2,45], potentially because of distracting the person sitting. As a result, it would appear sensible to combine pressure measurement with other objective information when evaluating sitting comfort/discomfort.

Beyond the controversy of how to sit comfortably, it is a challenge to distinguish different sitting postures in real-time. Firstly, pressure mats usually contain such large amounts of sensing elements (e.g., Tekscan 32 × 32 = 1024) that ideally require higher sampling frequencies (e.g., ADC unit) to acquire data with the minimal information loss. As a result, a compromise should be considered between higher resolution (more sensing elements) and the cost of hardware. To reduce the number of sensing elements, Xu et al. [64] developed a small sensor array (N = 256) which can achieve similar accuracy to commercial products. By converting pressure measurements to fidgeting movements, Cascioli et al. [48] reduced the number of pressure sensors to four and showed it was possible to resolve an association between discomfort and ICM. Secondly, processing large sensing information is time consuming. Finally, the recognition accuracy relies heavily on efficiency of algorithms. Though machine learning and neural networks have been applied, the accurate classification rate of eight different sitting postures is only 80% [51].

### 4.3. Objective Measurements Using Different Types of Instruments

In recent years, there have been some attempts to combine several different kinds of instruments (sensors and electronic devices) when exploring the effects of prolonged sitting on individuals. The devices used in these studies included electrocardiogram (ECG) [14], EMG (electrocardiogram) [63,65,86], IMU (Inertial Measurement Unit consisting of accelerometers, gyroscope and compass) [57,82,87,88], motion capture systems such as Vicon (Vicon Motion Systems Ltd., Oxford, UK) [87,89] and Optotrak (Northern Digital Inc, Ontario, Canada) [62,71] as well as infrared cameras [10,29].

By measuring blood flow, heart rate and body temperatures on legs and left tympanic membrane (core temperature), Hodges et al. [14] compared four types of wheelchair cushions and covers made of different materials and concluded that seat covers played an important role in sitting comfort. As lower-cost electronic chips with greater reliability become available, researchers have attempted to investigate the relationship between body movements and sitting comfort/discomfort by combining IMU, EMG and pressure mats [52,53,55,86,87]. Another instrument that has been used in the evaluation of sitting comfort is the motion capture system which can record body movements by attaching reflective markers on anatomical regions of interest [52]. Such multifactor measurement has been applied to many areas from office chairs [57,86] to car cushions [63] and surgery seats [65].

With the help of multiple sensors, sitting postures can be studied from lower limbs to upper bodies. In addition, the growth in available noninvasive wearable products (e.g., ActivPAL accelerometer, PAL Technologies, Glasgow) makes it possible to continuously monitor daily activities [55]. The acquired information will prove important for healthcare services and cushion purchases. As a result, such innovations should help develop strategies and self-help equipment that can help prevent pressure ulcer formation and improve the quality of life of patients. Furthermore, the fusion of information based on multiple sensors should help enhance the recognition of different sitting postures and serve as reliable feedback to seat designers. One example of this is the application of motion cameras, pressure mats and accelerometers to study an ergonomically redesigned truck seat (Force-3) during long haul driving, [52]. As a consequence of using this system, different sitting postures and body movements were found to be attributable to interface pressure changes. Comparing with the standard truck seat, the Force-3 was found to exhibit higher sitting comfort after two hours in their trials.

Accurately measuring sitting posture provides valuable and complementary information for medical professionals and physical therapists to prevent abnormal neuromuscular activities and biomechanical disorders [74,90,91]. Wearable IMUs have become an effective tool to gain reliable data related to human physical activities in daily life and to monitor sitting patterns which strongly affect comfort or discomfort for prolonged sitting [56,57].

Though measurement of multiple parameters can provide more sitting information, several disadvantages exist regarding the practical application. Firstly, using multiple devices increases the cost of the whole system, however this is not a significant barrier. Secondly, motion cameras can only be used in specific laboratory conditions and reflective markers attached to the participants interfere with “natural” body movements. In addition, existence and awareness of these markers may influence subjective perceptions such as comfort and discomfort. Thirdly, the mass, size and functional recording time of wearable electronics (e.g., IMU) rely on the embedded battery and electronic chips.

### 4.4. Reliability and Validity of Sensors

Although sensors in practical applications have been calibrated by manufacturers, it is necessary to verify their validity and reliability before conducting any measurement [28]. For example, McCarthy et al. [36] and Liu et al. [13,34] utilized traceably calibrated environmental chambers to study the accuracy and linearity of the sensors along with the associated repeatability and hysteresis. The reason for employing such caution is that the measuring range of commercially available sensors is usually broader than the practical microclimate measurement encountered in such experiments (e.g., temperature values at the body–seat interface usually vary between 20 °C and 35 °C, if users sit in a room with normal conditions [36]). Additionally, datasheets of sensors provide a general description of the product instead of one which is specific to the chip used in the experiment.

Regarding pressure sensors, it is critical to calibrate the whole system prior to carrying out any measurement, a suggestion endorsed by both the product manufacturers (in their manuals) and researchers [45,52]. Due to the sensitivity of materials forming pressure sensors, any bending or external force will cause deformation to the components. Consequently, the performance of the whole pressure measurement system must be calibrated before (and preferably after) conducting any trial [58].

### 4.5. Future Work

To avoid bias inherent in the subjective assessment methods, questionnaire-based sitting comfort or discomfort evaluation usually requires the study of a large population, which increases the cost and time consumption. In addition, environmental interaction [88], sitting time [84,92,93] and the task performed [94,95] were found to have influence on individual’s judgement and perceptions. As a result, objective measurement can not only serve as a useful tool but provide reliable feedback irrespective of external interference.

With the rapid development of modern technology, noncontact measurements have been applied to seat comfort/discomfort evaluation such as radiography [96], ultrasonography [97,98] and MRI [99,100,101]. After installing specific apps, smart phones could be turned into portable sitting posture recorders, which could be used to study motion as traditional products once did [102].

As the majority of the retrieved research works had recruited young healthy individuals, it will be necessary to include various population groups (e.g., old generation or wheelchair users) to derive more general conclusions. In addition, different seat structures and functions should be taken into account when measuring sitting comfort or discomfort. For example, wheelchair users are usually vulnerable to losing balance or being unable to adjust postures [10,15,54]. As a result, along with sitting comfort, support and protection are important for wheelchair design. As field tests showed that rough roads have negative influence on sitting comfort of drivers [35,37,70], vibration reduction has had to be considered when designing vehicle seats. Regarding comfort measurement of office chairs [57,86,96], adjustability of seat pan and back rest is usually critical as office workers usually have different anthropometry.

Though sitting comfort/discomfort study belongs to the field of ergonomics, it is also associated with many scientific areas such as electrical and electronic engineering, philology, psychology and biomedical engineering as well as medical and healthcare science. It may be better to diversify the composition of research teams by involving experts with different knowledge backgrounds.

## 5. Conclusions

The aim of this review was to study typical methods used to objectively measure the microenvironment changes at the body–seat interface. In addition, we also investigated the relationship between objective measurement and subjective evaluation on sitting comfort/discomfort. Though body–seat interface pressure was reported to correlate with perceived comfort/discomfort [2,3,4], other factors (e.g., temperature and relative humidity) should be taken into account when assessing the comfort/discomfort of prolonged sitting. Additionally, there was no consistency in terms of the relationship between various measured variables and subjective perception, probably due to the variations in experiment designs. So, it still appears necessary to determine the most influential factors capable of accurately reflecting the subjective feelings of comfort and discomfort after engaging in sedentary activities.

As a note of caution, although objective measurements can effectively monitor metabolic changes of the human body at the sitting interface and even aid in the development of more comfortable seating, sedentary activity is still going to be harmful to an individual’s health. Additionally, prolonged sitting can lead to endothelial dysfunction which is a biomarker of cardiovascular diseases [1,90]. So, it seems more important for end-users to avoid sedentary activities than to choose comfortable seats.

## Figures and Tables

**Figure 1:** Relationship between objective measurements of microenvironmental changes at the body–seat interface and the characteristics of seats (material and structure) and human (sitting activities and sitting duration). The characteristic factors influence subjective perception of sitting comfort or discomfort and can be measured with the help of electronic devices.

**Figure 2:** Flow chart of literature selection through the review phases. * Reference [15] includes both microclimate and pressure measurements; therefore, it was included in both categories. As a result, although the total number of included publications is *N* = 54, the sum of the two categories is greater (*N* = 37 + 18 = 55).

**Figure 3:** Summary of methods used to classify sitting postures which are believed to be associated with subjective sensations.

**Figure 4:** Comparison of different pressure measurement systems used in publications with respect to the number of sensors being utilized. Please note: those with large numbers of sensors are generally the “pressure mats”, discussed in the adjacent text.

**Table 1:** Overview of studies on microclimate measurements at the user-seat interface and subjective evaluation.

Author (Year)	Participant Information	Research Methodology	Objective Measurement	Subjective Evaluation **	Conclusions
Liu et al. (2019) [26]	Single healthy university student Height = 1.74 m Weight = 58 kg	Approach to the foam cushion at two different speeds (slowly or rapidly).	Three HTU21D (TE Connectivity Ltd., Rheinstrasse, Schaffhausen, Switzerland) sensors placed at left mid-thigh, right mid-thigh and coccyx.	N/A	Transient increase in RH at the onset of sitting was an artefact due to moisture from a warmer environment interacting with a colder sensor.
Havelka et al. (2019) [27]	*N* = 16 (detailed information not available due to commercial sensitivity)	60-min relaxation 180-min on-road driving 60-min break 180-min on-road driving (changeover between drivers and co-drivers) Compare the following seats: Seat 1 (standard): top–woven fabric (twill), middle–reticulated foam, bottom–jersey knitted layer Seat 2 (standard+): top—woven fabric (twill), middle–nonwoven, bottom–3D spacer knitwear	15 SHT21 (Sensirion AG, Staefa, Switzerland) sensors in five sequences with three sensors per row	Five-level Likert-type scale for comfort evaluation. Use the redefined subjective evaluation scoring system (4, 6, 8, 10) to better distinguish between categories.	Seat 2 had better thermal and ventilating performance than Seat 1. Possible to resolve differences between similar seat formulations.
Olney et al. (2018) [10]	*N* = 6 (M = 6, F = 0), wheelchair users with spinal cord injury at C5 or below Age = 60 ± 10.7 years BMI = 24.75 ± 3.58 kg/m^2^	100-min sitting on four wheelchair seating systems: (1) solid strap cushion (2) perforated strap cushion (3) foam cushion (4) air cell cushion	One capsule-shaped temperature-humidity integrated sensor (FH2, MSR Electronics GmbH, Seuzach, Switzerland) placed under the right medial thigh Infrared thermal camera (T450sc, FLIR Systems Inc., Wilsonville, OR, USA) measures heating and cooling characteristics three times: Preseating (room temperature), after 100-min sitting and 5 min after the subject being transferred out of the seat	N/A	Strap-based wheelchair cushions had better thermal emission capability as both solid and perforate strap-based seating systems cooled down faster than foam/air cell cushions when vacated. Based on the single point measurement at the skin-seat interface, no significant difference existed in RH.
Yang et al. (2018) [11]	*N* = 26 Age = 20–26 years BMI = 18.33–28.09 kg/m^2^	Two-hour sitting on two commercially available pressure-relief wheelchair cushions: (1) air-filled rubber cushion (2) foam-fluid hybrid cushion	Four SH15 (Sensirion AG, Staefa, Switzerland) attached to the skin fastened by a single strip of surgical tape at the locations of ischial tuberosities and thighs	N/A	Temperature significantly differed between the measured locations, while RH showed no significant difference.
Liu et al. (2018) [28]	*N* = 8 (M = 4, F = 4) Age = 23.6 ± 1.3 years Height = 1.69 ± 0.08 m Body mass = 56.2 ± 10.3 kg	20-min sitting on the following chairs: Chair 1: fabric cover + foam, Chair 2: wood, Chair 3: leatherette cover + foam	64 digital temperature sensors (18B20, Maxim Integrated, San Jose, CA, USA) forming an 8 × 8 thermal measurement matrix	Questions related to thermal comfort, for example, *“Did you feel any difference when sitting on the test chair compared to the chair used while you were waiting?”*	Created a sensor-array-based body–seat interface temperature measurement system. Thermal performance of three chair compositions were measured and compared without disrupting participants. Temperature field at the contact surface was not uniformly distributed
Sales et al. (2017) [29]	Single healthy participant	15-min sitting on eight types of chairs: *lyptus* wood, plywood, polypropylene, synthetic leather, melamine laminate, polyester fabric, metal and medium-density fibre board	RTD temperature probe (on the seat surface) Infrared camera (ThermaCAMP640, FLIR Systems Inc., Wilsonville, OR, USA)	N/A	All seats exhibited a higher cooling rate within the first five minutes of being vacated by participants. There was a significant variation at the beginning of cooling stage, but at the end of 15 min, all the seats reached environmental temperature, except for *lyptus* wood and plywood.
Pron et al. (2017) [30]	Single healthy participant Age = 34 years Height = 173 cm Body mass = 75 kg	35-min sitting on the honeycomb-structured cushion	CEDIP (CEDIP Infrared Systems, Croissy, Beaubourg, France) Titanium infrared camera (The first infrared image was taken on the upper side of the cushion, the second one on the lower side, and the last one on the canvas of the wheelchair)	N/A	Cushion structure had impact on heat loss and dissipation
Liu et al. (2017) [13]	*N* = 11 (M = 6, F = 5) Age = 21–40 years BMI = 19.31–26.44 kg/m^2^	20-min sitting on either foam or gel cushion	Three HIH4000 (Honeywell Co., Morristown, NJ, USA) sensors under the left mid-thigh, the right mid-thigh and coccyx	N/A	Different cushion materials had a significant effect on RH profiles at the body–seat interface
Hsu et al. (2016) [31]	*N* = 78 (M = 39, F = 39) Participants equally divided into three groups (*n* = 26) Group 1 Age = 21.9 ± 1.8 years BMI = 21.6 ± 2.8 kg/m^2^ Group 2 Age = 22.5 ± 2.4 years BMI = 22.2 ± 3.8 kg/m^2^ Group 3 Age = 22.2 ± 3.8 years BMI = 21.7 ± 2.1 kg/m^2^	Two-hour sitting on the following three cushions: air-filled rubber, foam–fluid hybrid and medium density foam	Skin temperature and RH were measured with four digital sensors (SH15, Sensirion AG, Staefa, Switzerland) placed under the ischial tuberosities and thighs bilaterally	N/A	Foam-fluid hybrid cushions exhibited the slowest temperature rise in comparison with standard foam and air-filled rubber cushions. No significant difference in RH between different cushions and RH reached a plateau during the two-hour sitting period.
Kumar et al. (2015) [32]	*N* = 10 (M = 0, F = 10) Age = 36.0 ± 5.56 years Height = 162.36 ± 5.57 cm Body mass = 65.59 ± 9.25 kg	25-min sitting on foam cushion	16 NTC-type medical grade sensors (General Electric Sensors, Fairfield, Connecticut, USA) placed around the ischial and thigh regions. (four on each ischial area, two on each thigh and two on skin-seat pan interface on each side)	Participants were allowed to adjust the temperature by regulating the seat air conditioning system. User’s self-selected comfort was attained when there was no further request for any change between two adjustment periods (5 min each).	Thermal comfort was achieved when the seating interface temperature was lower than the body temperature
Vlaovic et al. (2012) [33]	*N* = 6 (M = 3, F = 3) Age = 35 ± 4.3 years BMI = 23.9 ± 2.4 kg/m^2^	90-min sitting on the following office chairs: Model 1: A notch for coccyx and prostate, 2-layer ploy urethane Model 2: 3-layer ploy urethane Model 3: mobile in 3D, 2-layer ploy urethane Model 4: Mobile in all directions, 1-layer ploy urethane Model 5: Standard, 1-layer ploy urethane	Six S-THB-M008 (Onset Computer Corporation, Bourne, MA, USA) probes (three on seat surface, two in seat and one to monitor room conditions)	N/A	Seat surface temperature was always higher than its interior temperature. Surface moisture on a seat was different from that inside the seat.
Liu et al. (2011) [34]	*N* = 11 (M = 6, F = 5) Age = 21–40 years BMI = 19.3–26.4 kg/m^2^	20-min sitting on three seats: (foam, gel mould and solid wood)	Three temperature sensors (LM35, National Semiconductor Corporation, CA, USA) placed under left mid-thigh, right mid-thigh and coccyx	N/A	The significant difference between the three measurement locations indicated more sensors would be needed to accurately represent the thermal characteristics at the body–seat interface
Cengiz et al. (2009) [35]	*N* = 10 (M = 7, F = 3) Age = 30–34 years Height = 155–189 cm Body mass = 51–87 kg	60-min on-road driving while sitting on seats with either ramie blended seat cover or polyester seat cover	Skin temperatures (PAR Medizintechnik GmbH & Co. KG Sachsendamm, Berlin, Germany) recorded at four places (thigh, waist, back and right bottom) Skin wittedness (PAR Medizintechnik GmbH & Co. KG Sachsendamm, Berlin, Germany) recorded on the torso back	A seven-point scale for thermal sensation and four scale for body moisture	Subjective evaluation and objective measurements were positively correlated in terms of thermal comfort. Waist and back areas had the highest temperature values. Ramie blended seat covers were preferable to polyester seat covers due to reduced skin moisture and improved thermal regulation.
McCarthy et al. (2009) [36]	*N* = 10 (M = 5, F = 5) Age = 19–41 years BMI = 18.67–27.33 kg/m^2^	60-min sitting on foam cushions	Five LM35 temperature sensors (National Semiconductor Corporation, CA, USA) and five HIH4000 sensors (Honeywell Co., Morristown, NJ, USA) placed under front and middle parts of each thigh and ischia tuberosity	N/A	Various measurement positions showed different temperature and RH responses.
Cengiz et al. (2007) [37]	*N* = 10 (M = 3, F = 7) Age = 31.8 ± 2.2 years BMI = 22.95 ± 4.1 kg/m^2^	60-min on-road driving while sitting on three different seat covers (velvet, jacquard and micro fibre), respectively	Eight locations for temperature (PAR Medizintechnik GmbH & Co. KG Sachsendamm, Berlin, Germany) measurement (under thigh, inner thigh, stomach, side of body, chest, waist, back and right bottom) Two locations (torso front and torso back) for the skin RH (PAR Medizintechnik GmbH & Co. KG Sachsendamm, Berlin, Germany)	Seven-point scale for thermal sensation, four-point scale for body moisture, three-point scale for comfort on seat back and seat cushion and four-point scale for sweat level.	Three seat cover materials showed no significant difference in subjective thermal evaluation and objective temperature measurement. Objective measurement had a positive relationship with subjective evaluation. Skin wettedness on the posterior torso was significantly different across the three cushions, while skin wettedness on the anterior torso did not. Skin wettedness played more important role in comfort evaluation than skin temperature.
Stockton and Rithalia * (2007) [15]	*N* = 5 (M = 1, F = 4) Wheelchair users Age = 63.8 ± 15.1 years	10–16 h sitting (mean = 14.00, SD = 2.83 h) a day for continuous seven days. Four types of cushion: Airlite, Kombat, Primagel and Systam	Temperature and RH probes (Gemini Data Loggers, West Sussex, UK) inserted into the core of the cushion	Four-point scale comfort rating	Subjective sensation of comfort was not linked with temperature and RH.
Bartels et al. (2003) [38]	*N* = 4 (M = 4, F = 0) Mean age = 25 years Mean height = 177 cm Mean weight = 70 kg	180-min sitting on either leather cover + foam cushion or fabric cover + spacer knit cushion	Temperature and RH sensors (detailed information is not available)	Four-point scale for heat, moisture and comfort sensations.	Textile cover and cushion type can improve sitting comfort
Ferrarin and Ludwig (2000) [39]	A health male Age = 32 years Height = 185 cm Weight = 70 kg	15-min sitting on four cushions: silicone gel pad, air-filled rubber cells, gel-filled bubble and foam-filled bubble	Infrared camera (TVS-2000, Nippon Avionics Co., Tokyo, Japan)	N/A	Nonflat surface cushions (air-filled cells and bubble-shaped surfaces) showed lower peak temperatures than a flat surface cushion. Gel-filled bubble cushions had lower maximum temperatures than foam-filled bubble cushions. Temperatures at the thighs were higher than at the ischial regions.

M = male, F = female. RTD = Resistance Temperature Detector. NTC = Negative Temperature Coefficient. RH = Relative Humidity. * This article also applied pressure sensor and pressure-related contents were put into Table 2. ** In the 5th column, the comfort/discomfort scaling standards were listed. If the corresponding trial was not evaluated subjectively, the content would be indicated N/A (Not Applicable). All cited papers are presented in reverse chronological order.More than two thirds of the retrieved studies (13/18) were published in the past ten years (2010–2019), while only five articles appeared (5/18) in journals between 2000 and 2009, indicating an increasing interest in objectively measuring microclimate changes at the body–seat interface. Among these, seven papers (7/18) compared the objective results with a subjective assessment of comfort or discomfort perception using scale-rated questionnaires [15,27,37,38], self-selected thermal comfort [35] or asking questions related to subjective sensations [28,35].

**Table 2:** Overview of literature (listed in reverse chronological order) on pressure measurement at the body–seat interface where some studies compared the pressure information with subjective sensations.

Author (Year)	Participant	Measured Parameter	Seat Type	Sensor Unit	Subjective Evaluation	Conclusions
Mitsuya et al. (2019) [9]	*N* = 18 (M = 11, F = 7)	2D pressure map at the seat and backrest converted into 1D data	19 types of car seats	Pressure mat (LX100, XSENSOR Technology Co., Calgary, Alberta, Canada)	7-level score questionnaire included three aspects: scale feeling, body pressure feeling, and fitting feeling.	Subjective evaluation appeared strongly related to objective measurement. Body size and car seat types were associated with body pressure distribution.
Bontrup et al. (2019) [49]	*N* = 62 (M = 23, F = 40) Age = 43 ± 13 years Height = 170 ± 10 cm Body mass = 78 ± 21 kg;	Mean number of movements per working hour Mean number of positional changes per working hour Mean time period of stable sitting Percentage of transient periods during the whole working period	Call-centre office seat	Textile pressure mat (Sensomative GmbH, Rothenburg, Switzerland)	Questionnaire on acute and chronic low back pain. Chronic pain questionnaire consisted of two parts: Korff characteristic pain intensity and Korff disability. Acute pain questionnaire included: pain severity and pain-related interference of daily functions	Sitting behavior was associated with chronic back-pain. Seven sitting postures were studied (Upright, reclined, forward inclined, laterally tilted right/left, crossed legs right over left/left over right).
Fasulo et al. (2019) [50]	*N* = 25 (M = 13, F = 12) Age = 21.4 ± 0.5 years BMI = 22.3 ± 2.3 kg/m^2^	Centre of pressure	Classroom chair/combo desk (an hour test)	Sensor array (T&T medilogic Medizintechnik GmbH, Schönefeld, Germany)	5-point Likert scale Questionnaire on comfort and discomfort evaluation	The perceived lower-body comfort had a relationship with movement
Ahmad et al. (2019) [51]	*N* = 5 (F = 3, M = 2) Age = 33 ± 8 years Height = 180 ± 10 cm Body mass = 70 ± 21 kg	Total number of activated sensors Single sensing element values Sum of all sensing element values Average of sensing element values	Wheelchair	Flexible screen-printed piezo-resistive sensors (customized)	N/A	Cost-effective and flexible screen-printed sensors for large area pressure measurement. Four sitting postures (forward leaning, backward leaning, right leaning and left leaning) were recognized with an accuracy of 80%.
Cardoso et al. (2018) [52]	*N* = 20 (M = 10, F = 10) Age = 22.3 ± 2.16 years (M), 22.1 ± 0.8 years (F) Height = 179.4 ± 7.0 cm (M), 165.3 ± 7.27 cm (F) Body mass = 79.6 ± 11.3 kg (M), 61.1 ± 6.5 kg (F)	Peak pressure, average pressure, and centre of pressure trunk angle, neck angle and shoulder angle Lumbar spinal angle and thoracic angle	Two truck seats: a “Force-3” seat and “industry standard” seat	Xsensor (X2, XSENSOR Technology Co., Calgary, Alberta, Canada) pressure pad Four Optotrak motion capture cameras (Optotrak Certus, NDI Inc., Waterloo, Canada) Three triaxial accelerometers (ADXL320, Analog Devices, Norwood, Massachusetts, USA)	100 mm-scale RPD (ratings of perceived discomfort) and ASD (automotive seating discomfort) questionnaires	The Force-3 seat outperformed the industry standard seat. Reported to be due to adjustability in the seat height, pan length and backrest angle.
Worsley et al. (2018) [53]	*N* = 13 (M = 8, F = 5) BMI = 22.9 ± 2.7 kg/m^2^	Peak interface pressure Trunk movement Oxygen and carbon dioxide tensions	Leisure chairs with foam cushion and air cushion	Tekscan pressure mat (Tekscan Co., South Boston, MA, USA) Triaxial accelerometer (Shimmer Platform, Realtime Technologies Ltd., Dublin, Ireland) Transcutaneous gas electrodes (Model 841, Radiometer A/S, Denmark)	Five-point comfort score	Interface pressure and trunk movement provided information to remind sitters to adjust their positions during prolonged sitting. Bony prominences contacted with the cushions remained at risk during sedentary activities.
Li et al. (2017) [45]	*N* = 18 (M = 12, F = 6) Age = 23.89 ± 1.49 years BMI = 21.51 ± 2.92 kg/m^2^	Average contact pressure Mean peak pressure Mean contact area	Three different seat pitches (32 inches, 30 inches and 28 inches)	Two Tekscan (Tekscan Co., South Boston, MA, USA) thin-resistive- sensor pressure mats (seat pan and backrest)	Discomfort questionnaire using 5-point body part rating scale	The pitch of the seat and interface pressure had an impact on prolonged sitting comfort.
Ma et al. (2017) [54]	*N* = 12 (M = 7, F = 5) Age = 22–36 years BMI = 16–34 kg/m^2^	Mean and standard deviation Five sitting postures	Wheelchair	FSR (Interlink FSR-406, Interlink Electronics, CA, USA) sensors (seven on seat pan and 5 on backrest)	N/A	Compared five classification algorithms whereby the decision tree was capable of achieving an accuracy of 96.85%.
Stinson et al. (2017) [55]	*N* = 14 (M = 12, F = 2) patients with spinal cord injury (trial 1) N = 7 old patients (trial 2)	Interface pressure Trunk tilt angle	Wheelchair Hospital chair	X3 interface pressure mat (XSENSOR Technology Co., Calgary, Alberta, Canada) ActivPAL3 accelerometer (PAL Technologies, Glasgow, UK)	N/A	Interface pressure and body movement information facilitated occupational therapists and healthcare professionals to minimize the risk of developing sitting acquired pressure ulcers through correct interventions.
Ma et al. (2017) [56]	*N* = 12 (M = 7, F = 5) Age = 22–36 years BMI = 16–34 kg/m^2^	Centre of Pressure Angular velocities of anterior-posterior and medial-lateral swings	Wheelchair	FSR (Interlink FSR-406, Interlink Electronics, CA, USA) sensors (*n* = 6, equally placed on front, left/right and rear sides) IMU placed on the centre of the cushion (MPU9250, InvenSense Co., Tokyo, Japan)	N/A	Achieved an accuracy of (>89%) for activity recognition and (>98%) for activity level (quantified activity) recognition
Zemp et al. (2016) [57]	*N* = 41 (M = 25, F = 16) Age = 24–64 years Height = 160–200 cm Body mass = 53–126 kg	Median value of pressure Inclination angles of the backrest	Office chair	FSR (Interlink FSR-406, Interlink Electronics, CA, USA) sensors (n = 16, 10 on seat pan 4 on backrest, 2 on armrest)	N/A	The accuracy of classifying seven different sitting positions was between 81% and 98%.
Cascioli et al. (2016) [48]	*N* = 21 (M = 12, F = 9) Age = 25 ± 5 years Height = 1.73 ± 0.10 m BMI = 25 ± 4 kg/m^2^	In-chair movement (ICM)	Contoured foam Straight foam Wood	FSR (Interlink FSR-406, Interlink Electronics, CA, USA) sensors	Questionnaires using 11-point numerical rating scale	Discomfort was associated with increased ICMs, while fewer ICMs indicated increasing comfort.
Lee and Shin (2016) [40]	*N* = 7 (M = 2, F = 5) Age = 22 ± 0.58 years Height = 168.9 ± 6.57 cm Body mass = 59.14 ± 4.35 kg	Ratio of the average pressure	Office chair	Piezo-resistive conductive film sensor array (customized)	N/A	Pressure distribution was related with sitting posture (upright, forward leaning, and backward leaning)
Zemp et al. (2016) [41]	*N* = 20 (M = 13, F = 7) Age = 27–57 years Height = 1.60–1.89 m Body mass = 50–105 kg	Averaged movements of one working hour Averaged positional changes during one working hour Mean time period of stable sitting Mean duration in the same sitting positions Percentage of transient periods during the whole working time	Office chair	Pressure sensor mat (PST04, SensingTex, Barcelona, Spain)	Standardized questionnaires (KPI and BPI) were used to assess short and long-term back pain	Classification of seven sitting positions (upright, reclined, forward inclined, laterally tilted right/left, crossed legs right over left/left over right) with an accuracy >80% Subjects with slight back pain exhibited a more static sitting behavior compared to subjects without any discomfort
Zemp et al. (2016) [58]	*N* = 20 (M = 15, F = 5) Age = 20–37 years Height = 1.64–1.90 m Body mass = 52–99 kg	Peak pressure Mean pressure Standard deviation of the pressure distribution Total contact area Force Maximum pressure gradient Mean Pressure gradient Standard deviation of the pressure gradient	Nine office chairs	Two pressure mats (Pliance-x 32 Expert, Novel GmbH, Munich, Germany: seat pan and backrest)	N/A	The material properties of chairs strongly influenced pressure distribution.
Shu et al. (2015) [59]	A male subject Age = 30 years Height = 174 cm Body mass = 70 kg	Pressure value Contact area	90-min continuous working while sitting on office chairs	Textile resistive sensor arrays (customized)	N/A	The resistance matrix approach improved the measurement accuracy with lower hardware complexity and crosstalk error. Three sitting postures of sit-up, backward and forward were identified.
Fredericks et al. (2015) [60]	*N* = 201 (M = 100, F = 101) Age = 29.1 ± 11.1 years (M), 31.9 ± 12.4 years (F) Height = 1750.3 ± 77.9 mm (M), 1638.1 ± 69.6 mm (F) Body mass = 76.5 ± 13.1 kg (M), 66.8 ± 12.4 kg (F)	Standardized pressure map of seat pan and back rest	Customized chair with adjustable back rest support 15 min sitting while complete the task of typing/and using the mouse	FSA pressure mapping system (FSA Industrial Seat and Back Systems, Verg Inc., USA)	Optimal location and magnitude of backrest selected by users	Participants preferred asymmetric support in the lower back region which was contrary to popular practice
Barba et al. (2015) [61]	*N* = 9 Age = 59.7 ± 24.2 years Height = 1.76 ± 0.10 m Body mass = 38.78 ± 4.94 kg	12 posture recognition based on pressure values	Office chair	Customized piezo-resistive sensors (eight sensors on seat pan and eight on backrest)	N/A	Developed a simple and inexpensive hardware system to monitor different sitting postures
Yoo (2015) [62]	*N* = 10 (M = 10, F = 0) Age = 28.2 ± 3.9 years Height = 175.7 ± 4.7 cm Body mass = 68.1 ± 6.3 kg	Gluteal peak pressure Trunk flexion angle	A general chair A suspension seat support chair	TekScan system (Tekscan Co., South Boston, MA, USA)	N/A	Suspension seat support chair was shown to reduce pressure at gluteal and thigh areas and prevented a slumped sitting posture
Le et al. (2014) [63]	*N* = 12 (M = 6, F = 6) Age = 33.0 ± 13.4 years Height = 169.8 ± 9.5 cm Body mass = 69.2 ± 13.2 kg	Seat pan distribution Pan and back high pressure point percentages Pan and back oscillations EMG cycling muscle oxygenation	Car seats (Audi A8 seat and Chrysler Sebring seat)	Two piezoelectric X3 (XSENSOR Technology Co., Calgary, Alberta, Canada) pressure sensor mat (seat pan and seat back) EMG (Delsysw Inc., Bagnolie-16, Boston, MA, USA) Custom-made 16-channel near-infrared spectroscopy system	100mm-scale subjective discomfort for several body regions (neck, upper back, lower back, hip, buttock, upper leg and knee)	Body mass and stature had an impact on sitting discomfort.
Kyung and Nussbaum (2013) [42]	*N* = 22 (Y = 11, O = 11) Young group: Age = 21.8 ± 3.2 years Height = 168.9 ± 11.2 cm Body mass = 67.9 ± 11.1 kg Older group: Age = 71.4 ± 8.6 years Height = 168.2 ± 11.7 cm Body mass = 73.5 ± 22.0 kg	Contact area Contact pressure Peak pressure Ratio of local to global of contact area Ratio of local to global of contact pressure Ratio of local to global of peak pressure Local areas of seat: bilateral thighs and buttocks Local areas of seat back: low back and upper back	Two car seats (Sedan and Sport utility vehicle)	Two Tekscan pressure mats (Tekscan Co., South Boston, MA, USA)	Three subjective ratings (comfort, discomfort and overall). The comfort Scale ranged from 0 to 10, Whereas the discomfort scale ranged from 0 to −10.	Young and old subjects had different perceptions of comfort rating for the same car seats
Xu et al. (2013) [64]	*N* = 25 (M = 15, F = 10)	Canny edge detector Extract the outline curve of the binary image Measure the distance between every point and an image centre	Office chair	Customized textile pressure sensor (a fibre-based yarn coated with piezoelectric polymer)	N/A	The system appeared capable of resolving between seven sitting postures (sitting up, forward, backward, left lean, right lean, right foot over left and left foot over right) with an accuracy of 85.9% A resampling method reduced uncertain factors including offset, scaling, crosstalk and rotation effects
Noro et al. (2012) [65]	*N* = 11 (M = 7, F = 4) Height percentile information	Peak pressure Contact area Pelvic rotation	Two different surgery seats: a conventional seat and a prototype of a new seat (seat pan with sacral support)	Pressure sensitive mat (waiting for the corresponding author’s reply) Patented gyroscope (Patent no. 3,928,103 2004)	Five-point comfort rating	The newly designed chair was considered more comfortable than the traditional chair because it reduced the pressure and prevented posterior pelvic rotation
Paul et al. (2012) [66]	*N* = 64 (M = 64, F = 0) Age = 38 ± 6 years Height = 1730 ± 55 mm Body mass = 75.9 ± 11.7 kg	Contact areas (total seat, upper and lower seat back) Rear/front cushion force	Three vehicle seats	Tekscan (Tekscan Co., South Boston, MA, USA) sensor system	N/A	Anthropometric characteristics (e.g., body mass, shoulder breadth and hip circumference) were correlated with cushion contact areas and cushion front and rear force.
Meyer et al. (2010) [43]	*N* = 9 (M = 6, F = 3)	Centre of force Pressure at aggregated areas	Office chair	Customized textile pressure sensors	N/A	Classification accuracy for 16 sitting postures was almost the same as the commercially available products
Groenesteijn et al. (2009) [46]	*N* = 20 (M = 10, F = 10) Age = 43 ± 10.8 years Height = 1.77 ± 0.1 m Body mass = 75 ± 11.3 kg	Seat pan pressure: peak Pressure and pressure distribution	Office chair	Pressure sensitive mat (Pliance-x system, Novel Gmbh, Munich, Germany)	Six-point comfort rating	Comfort was related to task. Easily adjustable back rest was preferred by users.
Kyung and Nussbaum (2008) [67]	*N* = 27 (M = 12, F = 15) Age = 20–35 years Height = 170.7 ± 11.7 cm Body mass = 69.1 ± 13.1 kg	36 interface pressure variables (pressure levels, contact areas and ratios of local to global pressure)	Two car (sedan and SUV) + two seats + two test conditions (lab + field)	Two Tekscan (Tekscan Co., South Boston, MA, USA) pressure mat (seat and back)	Comfort and discomfort ratings of the whole body and six local parts. Rating scales ranged from 0 to −10, and from 0 to 10, for discomfort and comfort, respectively.	Pressure measurement was considered more suitable for short-time comfort/discomfort evaluation than long-term. Pressure ratios at buttocks were lower than for upper/lower back. 20 out of 36 pressure variables were correlated with either overall or whole body comfort ratings. No pressure variable had significant correlation with whole body discomfort.
Stockton and Rithalia * (2007) [15]	*N* = 5 (M = 1, F = 4) Wheelchair users Age = 63.8 ± 15.1 years	Mean ± SD	Four types of wheelchair cushions: Airlite, Kombat, Primagel and Systam	Interface pressure measured by Oxford Pressure Monitor II (Talley Group, Hants, UK)	Four-point scale comfort rating	Cushions with the lowest interface pressures were rated the most comfortable.
Carcone and Keir (2007) [44]	*N* = 30 (F = 15, M = 15) Age = 23 ± 3.1 years Height = 1.71 ± 0.09 m Body mass = 69.7 ± 15.3 kg	Mean of average pressure Mean peak pressure Mean contact area Centre of pressure	Office chair with different backrest pads	Capacitive pressure-sensing system (X236, XSENSOR Technology Co., Calgary, Alberta, Canada)	Five-point Likert scale.	Higher ranked backrest was associated with lower peak backrest pressure, greater seat pan contact area and smaller backrest area.
Vos et al. (2006) [68]	*N* = 24 (M = 12, F = 12)	Peak and average pressure Contact area	12 office chairs	X-Sensor pressure sensor mat (XSENSOR Technology Co., Calgary, Alberta, Canada) Four scales (under two arms and two feet)	N/A	Chair design had greater impact on sitting pressure than sitting posture, though both factors had significant relationships with pressure distribution.
Na et al. (2005) [69]	*N* = 16 (M = 16, F = 0) Age = 25.5 ± 2.6 years Height = 172.8 ± 5.4 cm Body mass = 72.3 ± 9.8 kg	Four body pressure ratio variables and two body pressure change variables	45-min simulated driving (15 laps of 3 min per lap) while sitting on mid-size sedan seat	FSR (FSA Industrial Seat and Back Systems, Verg Inc., USA) pressure mats (seat pan and back rest)	Seven-point comfort rating for six body parts (neck, shoulder, back, lumbar, hip and thigh)	Body pressure ratio variables can be used to evaluate driving posture. Body pressure distribution variables were associated with discomfort ratings.
Porter et al. (2003) [70]	*N* = 18 (M = 8, F = 10) Age = 40 ± 12 years	Mean and maximum interface pressure acquired from left and right ischial tuberosities, left and right thighs, upper back and lower back Eight angle parameters: ankle angle, arm flexion, elbow angle, knee angle, neck inclination, thigh from horizontal, trunk from vertical and trunk–thigh angle	Three types of cars equipped with two different seats on road trial	Capacitive sensor matrix (Novel, Munich, Germany) placed on seat and backrest Goniometer	Seven point discomfort rating	Interface pressure appeared to have no strong correlation with subjective discomfort during road trials.
Andreoni et al. (2002) [71]	*N* = 8 (M = 7, F = 1) Age = 25 ± 2 years Height = 1.80 ± 0.06 m Body mass = 74 ± 13 kg	Mean and peak pressures lumbar flexion angle	Car seat	Tekscan (Tekscan Co., South Boston, MA, USA) pressure mats (cushion and backrest) Motion cameras (Elite Image Inc., New York, NY, USA)	User self-selected comfortable position	Pressure sensor + motion capture were suitable to classify car driver postures
Hostens et al. (2001) [72]	*N* = 10 (M = 10, F = 0) Age = 26.5 ± 4.43 years Height = 174.98 ± 6.8 cm Body mass = 67.86 ± 8.9 kg	Maximum and mean buttocks Back support pressure	Four foam air-based seats for agricultural machinery	Capacitive pressure sensor (XSENSOR Technology Co., Calgary, Alberta, Canada) mats (seat and back rest)	Participants choose the most comfortable sitting position	A linear relationship presented between mean pressure and body mass index. The air-based seat had lower maximum pressure than the foam seat.
Brienza et al. (2001) [17]	*N* = 32 Age = 85 ± 7.6 years	Mean and peak pressure	Generic foam seat cushion and pressure-reducing seat cushion placed on wheelchair	Pressure sensitive mats (FSA Industrial Seat and Back Systems, Verg Inc., USA)	National Pressure Ulcer Advisory Panel staging method	Buttock-cushion interface pressure was associated with pressure ulcer development
Fenety et al. (2000) [73]	*N* = 8 (M = 1, F = 7) Age = 23–45 years Height = 158.5–170 cm Body mass = 59.3–85.5 kg	ICM centre of pressure	Working chair used by telecommunication directory assistance Operators for two hours	Force sensing resistors pressure mat (Force Sensing Systems, Winnipeg, MN, Canada)	Preferred chair and screen position were chosen by participants before trials	ICM and centre of pressure can represent objective sitting comfort/discomfort
Tewari and Prasad (2000) [47]	*N* = 3 Height = 164.5–172.5 cm Body mass = 51.4–75.5 kg	Mean pressure on the seat pan and back rest	Tractor seat (four back-rests with different radius and three back-rest inclination angles)	Pressure sensitive mats (waiting for the corresponding author’s reply)	General comfort 6-point scale	Lower mean pressures on the seat pan were associated with higher comfort scores.

M = male, F = female, FSR = force-sensing-resistor, BPI = Brief Pain Inventory, KPI = Korff Pain Inventory. * This article measured both microclimate and pressure information. As a result, it was placed in Table 1 and Table 2. IMU = Inertial Measurement Unit including a 3-axis gyroscope, a 3-axis accelerometer and a 3-axis digital compass.
